# Analysis of DAT Combined with the VSD Technique in Wound Repair of Rats and Its Effect on Inflammatory Factors

**DOI:** 10.1155/2022/2662876

**Published:** 2022-08-20

**Authors:** Xiaochen Sun, Chengxin Xu, Juan Lian, Mei Song

**Affiliations:** Department of Burns and Plastic Surgery, The 940th Hospital of Joint Logistics Support Force of Chinese PLA, Lanzhou 730050, China

## Abstract

The clinical efficacy of decellularized adipose tissue (DAT) combined with vacuum sealing drainage (VSD) in the treatment of wound healing in rats is investigated, and the changes of inflammatory factors are analyzed. The tissue defect model of SD (Sprague-Dawley) rats is established and divided into the combined group (*n* = 12) and the control group (*n* = 12) according to different treatment methods. The control group is treated with a single VSD technique, and the combined group is treated with DAT on the basis of the control group. The wound healing time of the two groups is observed. Wound tissue is collected 1 day, 10 days, 20 days, and 30 days after treatment, and neutrophil infiltration is observed by HE (hematoxylin-eosin) staining. The expression changes of IL-6 and IL-13 at each time point before and after treatment are compared. Histological observation shows that the cell infiltration is reduced in both groups, and the wound repair in the combined group is better than that in the control group. The experimental results show that the DAT combined with the VSD technique can further speed up wound healing and reduce inflammation in rats.

## 1. Introduction

With the continuous development of society, various industries and manufacturing industries are rising. The cases of soft tissue trauma and burn caused by accidents are increasing year by year. Tissue damage can expose subcutaneous muscles, nerves, and bones in a large area, which not only increases the risk of infection but also damages patients' aesthetics, seriously reduces patients' quality of life, and causes great psychological pressure [1, 2]. In the previous clinical repair of tissue trauma, traditional dressing change is mostly used for treatment, but this method could not meet the conditions required by the healing process of tissue trauma in patients and is prone to multiple complications. It had a poor effect on improving the prognosis of such patients and is no longer suitable for clinical practice [3]. However, with the continuous development of medical technology, vacuum sealing drainage (VSD), as an emerging technology for clinical treatment of wounds, can timely absorb secretions from the wound through negative pressure and provide excellent conditions for wound healing [4], while decellularized adipose tissue (DAT) has high histocompatibility and cell adhesion and has the ability to promote subcutaneous fat regeneration. However, current research studies on DAT mainly focus on adipose tissue engineering. There are relatively few studies on promoting tissue wound repair and healing [5, 6]. Therefore, this study established a tissue trauma model in SD (Sprague-Dawley) rats and discussed the application value of DAT combined with VSD technology to provide a theoretical basis for promoting and improving the prognosis of patients with wound defect in the future.

The rest of this paper is organized as follows: Section 2 discusses related work, followed by clinical data and the combined methods designed in Section 3.  Section 4 shows the experimental results and analysis, and Section 5 briefly summarizes all of standpoints of the whole text.

## 2. Related Work

Tissue defect is a common injury type after burns and car accidents. If the wound is not closed in time, the damaged tissue is exposed to the air for a long period, which will lead to the invasion of various microorganisms and pathogenic bacteria and then lead to various infectious complications, which will hinder the wound recovery and treatment in the later stage [7]. In the past, conventional debridement and dressing change were used in the treatment of tissue wound damage, which not only caused patients' pain but also increased the duration of dressing change with the extension of the severity of the wound, aggravating the psychological and physiological discomfort of patients [8]. With the wide application of VSD technology in clinical practice, it has been proved to have high clinical efficacy in the treatment of diabetic foot, ulcer wounds, etc. Numerous studies have shown that VSD can not only remove exudates and necrotic tissue in wounds in time but also reduce the infection rate to a certain extent [9]. The DAT structure has a variety of growth factors such as collagen, glycosaminoglycan, and VEGF, which can be used as a three-dimensional scaffold material to promote tissue regeneration. However, clinical studies have shown that it is easy to dry out and be polluted when applied alone to open wounds, further causing foreign body reaction and hindering wound healing [10]. All up, this study further explored the application value of DAT combined with VSD in wound repair of the rat skin defect model and laid a theoretical foundation for providing new treatment methods to accelerate wound recovery and improve prognosis of patients with tissue damage.

This study shows that the wound healing time of the combined group is shorter than that of the control group. After bleeding stops, wound healing needs four stages including inflammation, mature epithelial cell proliferation, organization, and inflammation. As one of the most important key points in this stage, if the inflammatory response cannot be controlled effectively and timely, it will cause the wound inside as the cell activity increases, induce a large number of proinflammatory factors, and inhibit tissue repair [11]. However, DAT combined with the VSD technique in the combined group could not only keep the wound surface clean and wet but also avoid the contamination of DAT dry junctions, maintain the biological activity of DAT during the treatment, improve the survival rate of fibroblasts, and further promote wound healing [12]. In addition, as the first defense response after trauma, inflammatory factors represented by neutrophils can rapidly secrete, proliferate, and gather near the wound surface to jointly resist the invasion of microorganisms and pathogenic bacteria, while IL-6 and IL-13 act as lymphatic factors between white blood cells and immune cells. They participate in hematopoietic and immune regulation together with blood cells and play an important role in regulating inflammatory response. When the expression level of IL-6 and IL-13 increases, it indicates the occurrence of inflammatory response in the body [13–15]. In this study, HE (hematoxylin-eosin) staining of neutrophils and ELISA detection of IL-6 and IL-13 levels showed that VSD combined with DAT could further reduce inflammatory response, reduce neutrophil infiltration, and promote rapid wound repair, and it indicated that adipocytes were the most expendable tissues in the human body. Adipocytes have the characteristics of wide source and the large yield, so removing such groups had no significant effect on the human body. At the same time, there is no fixed organization form of fat tissue; therefore, it contains a large amount of protein and the composition such as growth factors. Especially after cell-free processing operations, a lot of suitable substrate materials that are rich in protein and growth factors can be harvested for cell proliferation and migration. Aperture is suitable for cell growth, and it can promote stem cell differentiation, migration, and adhesion effects, promote the vascular endothelial cells in the lumen sample distribution, and accelerate wound healing. In this study, the healing speed and the decreased levels of inflammatory factors in Vanda-formed rats are consistent with those of the above theoretical mechanism [16, 17].

## 3. Clinical Data and Combined Methods

### 3.1. Modeling and Grouping of Rats

Twenty-four SPF male SD rats are randomly divided into the control group (*n* = 12) and the combined group (*n* = 12). They are purchased from the animal experimental center of 301 Hospital and fed with the same standardized feeding mode, which is approved by the Animal Ethics Committee. The abdominal skin of rats is disinfected with iodavor, and anesthesia is performed with 10% chloral hydrate. After the effect of anesthesia, a circular incision with a diameter of 10 mm is drilled in the back of rats, deep into the fascia layer. The skin and the anticontraction ring are sutured with 4-0 prolene line, and the sterile oil yarn is covered on the wound surface; the wound is wrapped with sterile dressing. Three anesthetics are randomly selected at T0, T1, T2, and T3 to observe the wound recovery, changes of inflammatory factors, and histological changes.

### 3.2. Combined Methods

#### 3.2.1. Treatment Methods

The control group uses VSD for debridement operation. First of all, for clear visible necrotic tissue and inflammatory granulation tissue, we use saline and iodine volts repeatedly for cleaning wounds, select VSD dressings that are similar to the size of wound, and cover the wound, which ensures good contact with dressings and the wound. They drained a silicone drainage tube 3 cm from the wound edge. The biological semipermeable film is covered outside the VSD dressing, and the adhesive range exceeds the edge of the VSD dressing by 5 cm. After the adhesive is firmly adhered, the central negative pressure is used for suction, with a negative pressure of -0.017 kPa∼0.06 kPa. After continuous suction for 7–14 d, the dressing could be removed and subsequent skin grafting could be carried out.

The combined group is combined with DAT on the basis of the control group. DAT is tiled on the wound surface before the CSD dressing is applied to the wound, and then, the VSD dressing is covered on the surface of DAT. Subsequent operations are the same as those in the control group.

#### 3.2.2. DAT Preparation Method

*(1) Sources of Adipose Tissue*. The adipose tissues in the experiment were all from the plastic and prosthetic department of our hospital. There were no large visceral lesions in adipose tissue, and the age was 18–35 years. Resource requirements: young healthy women, preoperative liposuction, and routine examination. Before liposuction, patients need to sign an informed consent form to identify the possible risks during the operation and agree to use adipose tissue samples. All liposuction fats come from the abdomen. During the operation, an injection needle with a diameter of 0.9 mm is used for anesthesia, and Liposuction technology for liposuction. The extracted fat is put into a sterilizing centrifugal tube for standby, and the excess fat is stored in a −80°C refrigerator for use.

*(2) Extraction, Passage, and Recovery of Human Adipose Stem Cells*. First, the fat granular tissue is cleaned and then cut into pieces with ophthalmic scissors. L-DMEM is added and then put into a constant temperature-shaking table for digestion for 40 min. The complete medium is added to terminate digestion, the filtrate is collected, and the supernatant is discarded after stratification, and the complete medium is added to precipitate cells for resuspension and inoculation in the Petri dish for the culture. The medium is replaced for the first time at 24 h and then every 48 to 36 h.

When the abundance of cells in the logarithmic growth phase reaches 90% in the Petri dish, the medium is discarded and PBS buffer is added for clarification. Then, trypsin digestion cells containing EDTA are added and placed under the microscope for observation. When the cells gradually become round and separated from the Petri dish, the reaction is terminated, and the Petri dish is repeatedly shaken to get the cells completely separated from the dish. After centrifugation, the supernatant and the culture medium are mixed to make cell suspension. 1 ml cell suspension is placed in a new Petri dish and placed in an incubator for observation.

The medium package containing polylysine is mostly culture dish. Thaw and store in a constant temperature water bath pipe in advance, wipe it clean, put it into a centrifuge tube containing complete culture medium, and centrifuge it for 5 min. After the supernatant was added to the configuration, the medium suspension cells, the suspension cells in the culture dish, and the adherent cells in the incubator were observed. Decide whether to change the fluid according to the cell apoptosis.

*(3) Preparation of DAT*. In this paper, the fat in the centrifuge tube was repeatedly washed with sterile PBS for 3 times, and the swelling in blood and body fluid was eliminated after repeated beating and mechanical emulsification with nano fat cutter for 30 times. In this paper, the fat was repeatedly frozen and thawed for 3 times with a mesh filter, and then centrifuged in a centrifuge for 3 minutes to remove the upper oil and the lower sediment. EDTA containing trypsin is added and shaken overnight in an incubator. We wash it with sterile PBS 3 times, 30 min each; 99.9% isopropyl alcohol is treated for 36 h and replaced every 12 h; sterile PBS is washed 3 times, 30 min each time, and 0.25% trypsin is added and treated in a 37°C, 120rMP constant temperature culture shaker for 4 h. The obtained adipocyte extracellular matrix is placed on a well plate, stored overnight in a cryogenic box at −80°C, and lyophilized in a vacuum lyophilizer for 24 h before being sealed for use. All acellular fluids are treated with 1% penicillin/streptomycin and PMSF in a 37°C, 120rmp constant temperature incubator.

*(4) Microscopic Observation*. The DAT material is placed in a Petri dish and soaked in PBS for 24 h. The surface of the DAT material is observed under a microscope and photographed at different intervals. The ultrastructure is fixed with 2.5% glutaraldehyde overnight, washed by PBS for 2-3 times, dehydrated by gradient ethanol, soaked in iso-amyl acetate, and observed by a scanning electron microscope.

#### 3.2.3. Detection of IL-6 and IL-13 by ELISA

At each time point before and after treatment, 5 ml of fasting venous blood is taken from the patients in the morning and centrifuged for 10 min at a speed of 3500 r/min. The supernatant is taken after centrifugation, and serum IL-6 and IL-13 are detected by the ELISA. The kits are purchased from Shanghai Enzyme-linked Biotechnology Co., LTD. The instructions are followed as per the manufacturer's kit.

#### 3.2.4. Histological Observation by HE Staining

The wound tissues of the two groups of patients were observed at various time points before and after treatment. After acute washing, they were fixed in 4% paraformaldehyde with PBS solution, embedded in paraffin for about 24 hours, and cut into thin slices with a thickness of 8 um. After the HE staining method is adopted to improve the dyeing under observation of an electron microscope, we adjust the lens view of 400 x, 8 fields are randomly selected from each section, and the morphologic identification and counting of neutrophils within the field are performed, and the mean value is taken.

### 3.3. Statistical Treatment

SPSS 25.0 statistical software is used for data analysis. There are three steps as follows. (1) Measurement data: The normality test is performed on the data first. If the data follow normal distribution and homogeneity of variance, they are represented by the mean ± standard deviation. The paired sample *T test* is used for testing within the group, variance comparison is used between the groups, and repeated measurement analysis of variance is used between multiple groups, and the spherical test is performed. (2) Counting data are expressed in percentage, and the *x*2 test is performed. (3) Univariate and multivariate analysis of risk factors for post-treatment infection in the combined group is performed. *P* < 0.05 indicates significant difference.

## 4. Experimental Results and Analysis

### 4.1. Preparation Results and Microscopic View of the DAT Material

Figure 1 shows the DAT material prepared in this study. Figures 2 and 3 show the observation of the structure of the DAT material under an electron microscope and a light microscope, and it can be seen from Figures 1–3 that the structure is loose and porous; the DAT material still maintains its original shape after immersing in PBS, without dispersion.  Figure 4 shows the result of HE staining, and it can be seen from Figure 4 that DAT has no obvious cell structure, which suggests that the decellularization is complete.

### 4.2. Wound Healing Time

Table 1 shows the comparison of hospital indicators. It can be seen from Table 1 that the postoperative wound healing time and hospitalization time in the combined group are significantly lower than those in the control group (all *P* < 0.05).

### 4.3. Histological Changes and Neutrophil Count at Each Time Point after Treatment

Table 2 shows the value changes in the neutrophil count. In Table 2, “*∗*” means that compared with T0, *∗P* < 0.05; “#” indicates that compared with T1, #*P* < 0.05; “&” means & *P* < 0.05 compared with T2.  Figure 5 shows the changes in the neutrophil count. In Figure 5, “*a*, *b*, *c*, *d,*” respectively, means that if the same letter is shared between groups, *P* > 0.05 at different time points; “#” indicates that *P* < 0.05 between the two groups compared at the same point. Through the above experimental results, it can be observed that the neutrophil counts in both groups are lower after treatment than before, and neutrophil counts in the combined group are lower than those in the control group at each time point after treatment (*P* < 0.05).  Figure 6 shows the changes of wound tissue staining at each time point after treatment in the combined group.  Figure 7 shows the changes of wound tissue staining at each time point after treatment in the control group. It is clearly evident from Figures 6 and 7 that the cell infiltration is reduced in both groups, and the wound repair in the combined group is better than that in the control group.

### 4.4. The Expression Changes of IL-6 and IL-13 at Each Time Point before and after Treatment

The expression of IL-6 in each group is shown in Table 3 and Figure 8, and the trend of IL-13 is shown in Table 4 and Figure 9. In Tables 3 and 4, “*∗*“ means that compared with T0, *∗P* < 0.05; “#” indicates that compared with T1, #*P* < 0.05; “&” means & *P* < 0.05 compared with T2. In Figures 8 and 9, “*a*, *b*, *c*, *d,*” respectively, means that if the same letter is shared between groups, *P* > 0.05 at different time points; “#” indicates that *P* < 0.05 between the two groups compared at the same point. Through the above experimental results, it can be observed that before treatment, there is no difference in the expression of IL-6 and IL-13 in the two groups, but after certain treatment, the expression of all inflammatory factors is decreased, and the inflammatory factors in the combined group are lower than those in the control group at each time point after treatment (all *P* < 0.05).

## 5. Conclusion

The clinical efficacy of DAT combined with VSD in the treatment of wound healing in rats is investigated, and the changes of inflammatory factors are analyzed. The application of VSD combined with DAT in the repair of tissue damage can further accelerate the wound healing speed, reduce the pain sensation, and reduce the body's inflammatory response. This study can lay a solid theoretical foundation for the clinical application of tissue defect repair in the future.

## Figures and Tables

**Figure 1:** DAT materials of different shapes and sizes.

**Figure 2:** Observation under the electron microscope.

**Figure 3:** Observation under the light microscope.

**Figure 4:** HE staining results.

**Figure 5:** Changes in the neutrophil count.

**Figure 6:** Changes of wound tissue staining at each time point after treatment in the combined group: (a) T1; (b) T2; (c) T3.

**Figure 7:** Changes of wound tissue staining at each time point after treatment in the control group: (a) T1; (b) T2; (c) T3.

**Figure 8:** IL-6 changes.

**Figure 9:** IL-13 changes.

**Table 1:** Comparison of hospital indicators.

Group	*n*	Wound healing time
Control group	12	21.14 ± 3.31
Combined group	12	14.44 ± 2.64
*t*		13.796
*P*		<0.001

**Table 2:** Value changes in neutrophil count.

Group	*n*	*T*0	*T*1	*T*2	*T*3	*F*	*P*
Combined group	12	39.93 ± 4.14	27.72 ± 3.35*∗*	16.63 ± 2.25*∗*^#^	9.53 ± 1.42*∗*^#&^	7.723	<0.001
Control group	12	39.72 ± 4.08	30.36 ± 3.85*∗*	22.35 ± 2.73*∗*^#^	11.74 ± 1.46*∗*^#&^	5.624	<0.001
*t*		0.315	−4.510	−14.095	−9.460		
*P*		0.753	<0.001	<0.001	<0.001		

**Table 3:** The trend of IL-6 changes.

Group	*n*	T0	T1	T2	T3	*F*	*P*
Control group	12	26.35 ± 3.32	21.23 ± 2.21*∗*	16.63 ± 1.73*∗*^#^	12.22 ± 1.12*∗*^#&^	7.742	<0.001
Combined group	12	26.28 ± 3.29	18.83 ± 2.04*∗*	12.34 ± 1.24*∗*^#^	9.44 ± 1.03*∗*^#&^	11.245	<0.001
*t*							
*P*							

**Table 4:** The trend of IL-13 changes.

Group	*n*	T0	T1	T2	T3	*F*	*P*
Control group	12	36.63 ± 3.25	32.74 ± 2.86*∗*	29.35 ± 2.78*∗*^#^	26.63 ± 2.32*∗*^#&^	5.723	<0.001
Combined group	12	36.66 ± 3.19	30.22 ± 2.74*∗*	24.42 ± 2.53*∗*^#^	20.16 ± 2.15*∗*^#&^	8.624	<0.001
*t*		0.046	−4.454	−9.181	−14.318		
*P*		0.963	<0.001	<0.001	<0.001		

## Data Availability

The simulation experiment data used to support the findings of this study are available from the corresponding author upon request.

## References

[1] Wilkinson H. N., Hardman M. J. (2020). Wound healing: cellular mechanisms and pathological outcomes. *Open Biology*.

[2] Jiang D., Rinkevich Y. (2021). Furnishing wound repair by the subcutaneous fascia. *International Journal of Molecular Sciences*.

[3] Xue X., Li N., Ren L. (2021). Effect of vacuum sealing drainage on healing time and inflammation-related indicators in patients with soft tissue wounds. *International Wound Journal*.

[4] Ren L., Zhang C., Zhao L., Li C., Zhang L., Xue X. (2021). Influence of incentive nursing intervention on recovery of burn patients after vacuum sealing drainage. *International Wound Journal*.

[5] Mohiuddin O. A., Campbell B., Poche J. N. (2020). Decellularized adipose tissue: biochemical composition, in vivo analysis and potential clinical applications. *Advances in Experimental Medicine & Biology*.

[6] Yang J. Z., Qiu L. H., Xiong S. H. (2020). Decellularized adipose matrix provides an inductive microenvironment for stem cells in tissue regeneration. *World Journal of Stem Cells*.

[7] Monavarian M., Kader S., Moeinzadeh S., Jabbari E. (2019). Regenerative scar-free skin wound healing. *Tissue Engineering Part B Reviews*.

[8] Veith A. P., Henderson K., Spencer A., Sligar A. D., Baker A. B. (2019). Therapeutic strategies for enhancing angiogenesis in wound healing. *Advanced Drug Delivery Reviews*.

[9] Huang Q., Huang K., Xue J. (2021). Vacuum sealing drainage combined with free anterolateral femoral skin flap grafting in 16 cases of pediatric soft tissue damage to the foot and ankle. *Translational Pediatrics*.

[10] Robb K. P., Juignet L., Morissette Martin P. (2021). Adipose stromal cells enhance decellularized adipose tissue remodeling through multimodal mechanisms. *Tissue Engineering Part A*.

[11] Jiang X., Lai X. R., Lu J. Q., Tang L. Z., Zhang J. R., Liu H. W. (2021). Decellularized adipose tissue: a key factor in promoting fat regeneration by recruiting and inducing mesenchymal stem cells. *Biochemical and Biophysical Research Communications*.

[12] Chun S. Y., Lim J. O., Lee E. H. (2019). Preparation and characterization of human adipose tissue-derived extracellular matrix, growth factors, and stem cells: a concise review. *Tissue Engineering and Regenerative Medicine*.

[13] Xia Z., Guo X., Yu N. (2020). The application of decellularized adipose tissue promotes wound healing. *Tissue Engineering and Regenerative Medicine*.

[14] Leclerc C. J., Cooper T. T., Bell G. I., Lajoie G. A., Flynn L. E., Hess D. A. (2021). Decellularized adipose tissue scaffolds guide hematopoietic differentiation and stimulate vascular regeneration in a hindlimb ischemia model. *Biomaterials*.

[15] Han T., Walker J., Grant A., Dekaban G., Flynn L. (2021). Preconditioning human adipose-derived stromal cells on decellularized adipose tissue scaffolds within a perfusion bioreactor modulates cell phenotype and promotes a pro-regenerative host response. *Frontiers in Bioengineering and Biotechnology*.

[16] Ladhani H. A., Young B. T., Posillico S. E. (2021). Risk factors for wound infection in outpatients with lower extremity burns. *The American Surgeon*.

[17] Shettigar K., Murali T. S. (2020). Virulence factors and clonal diversity of *Staphylococcus aureus* in colonization and wound infection with emphasis on diabetic foot infection. *European Journal of Clinical Microbiology & Infectious Diseases*.

